The article "Analysis of Coagulation Abnormality in Patients with Multiple Myeloma and Its Clinical Significance" was retracted in 2023. Reasons: unreliable results or conclusions; concerns about the data; concerns about the peer review; concerns about the citations.

# Analysis of Coagulation Abnormality in Patients with Multiple Myeloma and Its Clinical Significance

**DOI:** 10.1155/2022/5120967

**Published:** 2022-06-20

**Authors:** Pengji Pan, Junxia Liu

**Affiliations:** ^1^Department of Hematology, Yongchuan Hospital of Chongqing Medical University, Chongqing 402160, China; ^2^Department of Oncology, Yongchuan Hospital of Chongqing Medical University, Chongqing 402160, China

## Abstract

**Objective:**

To analyze the abnormal changes of coagulation indexes in patients with multiple myeloma (MM) and their clinical significance on prognosis.

**Methods:**

Among 80 patients with MM, there were 24 patients of light chain type, 36 patients of IgG type, and 20 patients of IgA type. In the same period, 30 healthy people were in the control group. The laboratory indexes such as plasma prothrombin time (PT), activated partial thromboplastin time (APTT), fibrinogen (FIB), thromboplastin time (TT), D-dimer (D-D), and platelet (PLT) were detected and compared. The prognosis of MM patients was followed up, and the effects of various coagulation indexes on the prognosis of MM were analyzed by single-factor and multifactor analyses.

**Results:**

The PT and APTT of IgG and IgA groups were longer than those of the control group and the light chain group (*P* < 0.05), but there was no significant difference between the IgG group and the IgA group, the control group, and the light chain group. There was no significant difference in FIB values among the four groups (*P* > 0.05). The D-D content in the light chain group was higher than that in the control group, the IgG group, and the IgA group (*P* < 0.05). During the follow-up period, of 80 MM patients, 61 patients survived and 19 patients died. Univariate analysis showed that APTT, PT, and D-D were the factors affecting the prognosis of MM patients, and the differences were statistically significant (*P* < 0.05). Multivariate analysis showed that PT was an independent factor affecting the prognosis of MM patients (*P* < 0.05). *Discussion*. Patients with MM have clotting abnormalities. Patients with IgA and IgG type MM have a longer clotting time than patients with other types of MM, and patients with light-chain type MM have higher D-D content and are more prone to thrombosis. PT is an independent factor affecting the prognosis of MM patients, and analysis of coagulation abnormalities is important for evaluating the prognosis of patients.

## 1. Introduction

Multiple myeloma (MM) is a kind of hematological malignant tumor caused by the malignant clonal proliferation of terminal B lymphocytes, namely, plasma cells. The abnormal increase of monoclonal immunoglobulin or light chain is the main serological manifestation [1, 2]. It mainly occurs in the elderly, but in recent years, it has a tendency to be younger. Because the onset of the disease is hidden and the clinical manifestations are diverse, it is often misdiagnosed at the first diagnosis [3]. The most important pathological features of MM patients are the abnormal proliferation of monoclonal plasma cells in the bone marrow, secretion of a large amount of monoclonal immunoglobulins (M protein), and the deposition of M protein in related tissues or organs, resulting in corresponding injuries, such as multiple osteolysis, abnormal blood loss, and kidney injury [4, 5]. Among them, abnormal coagulation is the main cause of death in patients with multiple myeloma, which seriously affected the patients' health and quality of life [6].

The pathological basis of hemorrhage in patients was vascular endothelial cell injury and fibrinolytic-coagulation system dysfunction [7]. At present, clinically, it is believed that the mechanism of abnormal blood coagulation in MM patients may be that M protein can specifically inhibit the activity of various blood coagulation factors, which leads to the inhibition of blood coagulation function [8]. Tumor can invade blood vessel wall and promote the release of procoagulant factors from blood vessel wall. In addition, tumor cells metastasize and invade tissues and organs, resulting in tissue damage and endothelial cell damage. After endothelial cell injury, a large number of tissue factors can be released to activate the body's coagulation system, which then leads to coagulation-fibrinolysis dysfunction in patients [9, 10]. D-dimer (D-D), fibrinogen (FIB), prothrombin time (PT), etc. are all important indexes reflecting the body's coagulation function [11]. Some studies have shown that compared with normal people, MM patients have abnormal coagulation, but there is no systematic report on the characteristics of coagulation indexes of different types of MM patients [12]. In this study, the abnormal changes of coagulation indexes of MM patients and their clinical significance for prognosis were further analyzed by detecting various coagulation indexes of MM patients in our hospital and following up the prognosis of patients.

## 2. Materials and Methods

### 2.1. Subjects

A total of 80 MM patients from January 2020 to December 2021 in the Department of Hematology in our hospital were selected. In the same period, 30 healthy people were in the control group. Inclusion criteria: the diagnosis was made by bone marrow, immunology, and cytology; coagulation function is normal, no blood diseases; and complete data of cooperation and follow-up. Exclusion criteria: patients with serious cardiovascular and cerebrovascular diseases; major surgery in the near future or taking drugs that affect coagulation; and hemophilia, vitamin K deficiency, traumatic coagulation disorder, and other diseases that can lead to elevated globulin. According to the serum M components, MM patients were divided into three groups: the light chain group (*n* = 24), IgG group (*n* = 36), and IgA group (*n* = 20). This study was approved by the ethics committee of our hospital, and the patients and their families were informed and agreed.

### 2.2. Methodology

The venous blood of the patient was collected in a heparin anticoagulation tube and a sodium citrate (3.2%) anticoagulation tube and then centrifuged at 3000 r/min for 10 min with a Xiangyi TDZ5-WS centrifuge. The plasma thromboplastin time (TT), PT, activated partial thromboplastin time (APTT), FIB, D-D, and platelet (PLT) of the subjects were measured, respectively. The above reagents were purchased from Johnson & Johnson and Siemens, respectively. The reference range of PT is 9.00–13.00 s; the reference range of APTT is 20.00–40.00 s; the reference range of FIB is 2.00–4.00 g/L; the reference range of TT is 14.00–21.00 s; the reference range of D-D is 0.00–0.55 *μ*g/mL; and the reference range of PLT is 100–400 × 10^9^/L.

The prognosis of MM patients was followed up until January 2022. The single-factor and multi-factor analyses of the impact of various coagulation indicators on the prognosis of MM were conducted.

### 2.3. Statistical Analysis

Data analysis was performed using SPSS 23.0 statistical software. All study data were in accordance with the normal distribution. Measurement results such as age, TT, PT, APTT, FIB, D-D, and PLT level were expressed as the mean standard deviation ($\bar{x}$ ± *s*), and *t* test was used for comparison. The counting data such as gender and DS stage were tested by *χ*^2^ test. Logistic regression analysis was used to analyze the multiple factors influencing the prognosis of MM patients. *P* < 0.05 indicated that the difference was statistically significant.

## 3. Result

### 3.1. Comparison of General Information among Groups

There were no significant differences in general information such as gender and age among the control group, the light chain group, the IgG group, and the IgA group (*P* > 0.05), as shown in Table 1.

### 3.2. Comparison of Coagulation Indicators among Groups

The PT and APTT were longer in the IgG group and the IgA group than in the control group and the light-chain group (*P* < 0.05), but there were no significant differences between the IgG group and the IgA groups, the control group, and the light chain group. There was no significant difference in FIB values among the four groups (*P* > 0.05), as shown in Figures 1–3.

### 3.3. Comparison of Anticoagulant and Fibrinolytic System Related Indicators among Groups

The D-D content in the light chain group was higher than that in the control group, the IgG group, and the IgA group (*P* < 0.05), but the difference between the IgG group and the IgA group was not statistically significant (*P* > 0.05), as shown in Figures 4–6.

### 3.4. Univariate Analysis of Prognosis of Patients with MM

During the follow-up period of 80 MM patients, 61 patients survived and 19 patients died. Univariate analysis of the age, gender, coagulation indicators, and other clinical indicators showed that APTT, PT, and D-D were the factors affecting the prognosis of MM patients, and the differences were statistically significant (*P* < 0.05), as shown in Table 2.

### 3.5. Multifactor Analysis of Prognosis of MM Patients

Further multivariate analysis of APTT, PT, and D-D revealed that PT was an independent factor affecting the prognosis of MM patients (*P* < 0.05), as shown in Tables 3 and 4.

## 4. Discussion

Plasma cells in MM patients' bone marrow proliferate uncontrollably and produce monoclonal Ig, or M protein. After serum fixation and electrophoresis, the M protein of MM patients could be divided into light chain type, IgG type, IgA type, etc. The heavy chains of abnormal Ig synthesized and secreted by MM are different, but the light chains have only *κ* or *λ* forms and present a single increased light chain [13, 14]. The diagnosis and typing of MM is mainly based on the evaluation of M protein content in serum or urine by electrophoresis or immunofixation and free light chain analysis [15]. A total of 80 MM patients were included in the study. According to the serum M content of patients, they were divided into the light chain group (*n* = 24), IgG group (*n* = 36), and IgA group (*n* = 20).

In tumor patients, blood is hypercoagulable and one or more coagulation indexes are abnormal, which is more common in MM patients [16]. Papageorgiou et al. proposed that MM, as the most common progressive malignant tumor in plasma cell disease, has a prognosis ranging from several months to several years, and hypercoagulable state is a common hemodynamic change in newly diagnosed patients [17]. At home and abroad, there is little research on the correlation between coagulation level monitoring and the prognosis of MM. In this paper, the coagulation index levels and related clinical data of MM patients were statistically analyzed. The results show that the PT and APTT of the IgG group and the IgA group were longer than those of the control group and the light chain group, but there was no significant difference between the IgG group and the IgA group. It indicated that APTT and PT abnormalities were more common in patients with IgG and IgA, which was consistent with the results of Huang et al. [18]. This indicates that IgA and IgG types are more likely to cause abnormal coagulation system in MM patients than light chain types, which may be because IgG and IgA immunoglobulin are easy to combine with themselves to form polymers. And IgG and IgA immunoglobulin can combine with coagulation factors or other plasma proteins in plasma, causing high viscosity at low concentration, thus inducing hemorrhage. In addition, M protein can cover platelets and coagulation factors and affect platelet aggregation, thus interfering with the normal coagulation process, resulting in abnormal coagulation [19, 20].

D-D is a characteristic molecular marker of degradation of cross-linked fibrin under the action of a fibrinolytic enzyme, and it only increased in plasma during thrombosis. It is characterized by good stability, high sensitivity, and strong specificity (citation) [21]. In this study, the D-D content of different groups was compared, and it was found that the D-D content of the light chain group was significantly higher than that of the control group, the IgG group, and the IgA group in MM patients. It indicated that patients with MM had a tendency to form thrombus, and D-D abnormalities were more common in light-chain MM patients. Patients with light chain MM were more likely to form thrombus. High expression of MM cells means that microbubbles with anticoagulant effects contain a high concentration of substances that affect mesenchymal and endothelial cell antigen factors and induce cell migration and proliferation through specific signal transduction pathways, thus increasing endothelial cell thrombosis [22]. This may explain the fact that the incidence of thromboembolism events in MM is higher than that in normal people, and the plasma thrombomodulin and D-D levels in MM are higher than those in normal people [14].

Elyamany et al. found that tumor patients have coagulation dysfunction and the risk of thrombosis was increased [23]. The occurrence of thrombosis was easy to cause the occurrence and metastasis of tumors, indicating that coagulation abnormalities were correlated with tumor prognosis. In addition, it is suggested that the evaluation of coagulation function can predict the prognosis and disease progression of MM patients [24]. As one of the common tumors in the hematology department, MM has coagulation abnormalities such as hypercoagulability and hemorrhage, but there are few related studies on the prognosis of MM patients. In this study, 80 patients with MM were followed up for a long time. During the follow-up period, 61 patients survived and 19 died. Univariate analysis showed that the prognosis of MM patients with abnormal APTT, PT, and D-D was poor. To confirm the significance of coagulation dysfunction in the prognosis of MM patients. Further multivariate analysis showed that PT was an independent factor affecting the prognosis of MM patients. It is suggested that coagulation indexes have some influence on the survival rate and follow-up results of patients. The function of coagulation is closely related to the invasion and migration of tumor cells. Tumor cells need a large amount of blood supply in the process of proliferation and migration, which greatly interferes with the coagulation function of the body [25, 26]. The risk assessment of thrombosis in MM patients is valuable for the prognosis and curative effect assessment of MM patients, which further illustrates the role of the detection of relevant coagulation indexes in the prognosis of MM.

There are still some deficiencies in our study. This study only compared the coagulation functions of different types of MM patients, and the correlation between the coagulation functions of MM patients and various clinical indexes needs further observation in follow-up studies. In addition, the number of cases included in the study is small, so it is necessary to accumulate more cases to further explore the mechanism of coagulation abnormality in MM patients.

In summary, among the different types of MM, IgA type and IgG type MM are more likely to affect the coagulation system, and compared with the IgA type and IgG type MM, the light chain type is more likely to form thrombus. Analysis of abnormal blood coagulation plays an important role in evaluating the prognosis of patients and provides the basis for adopting correct clinical strategies and timely intervening in severe complications.

## Figures and Tables

**Figure 1:** Comparison of PT values between groups. Note: compared with the control group, ^*∗*^*P* < 0.05; compared with the light chain group, ^#^*P* < 0.05.

**Figure 2:** Comparison of APTT values among groups. Note: compared with the control group, ^*∗*^*P* < 0.05; compared with the light chain group, ^#^*P* < 0.05.

**Figure 3:** Comparison of FIB values among groups.

**Figure 4:** Comparison of TT values among groups.

**Figure 5:** Comparison of D-D values among groups. Note: ^*∗*^*P* < 0.05, compared with the light chain group.

**Figure 6:** Comparison of PLT values among groups.

**Table 1:** Comparison of general information among groups.

Group	Gender		Age (years)	DS staging		
	Male	Female		I	II	III
Control group (*n* = 30)	18 (60.00%)	12 (40.00%)	57.82 ± 6.94	—	—	—
Light chain group (*n* = 24)	16 (66.67%)	8 (33.33%)	56.91 ± 7.05	4 (16.67%)	4 (16.67%)	16 (66.67%)
IgG group (*n* = 36)	23 (63.89%)	13 (36.11%)	58.62 ± 6.51	3 (8.33%)	6 (16.67%)	27 (75.00%)
IgA group (*n* = 20)	11 (55.00%)	9 (45.00%)	58.14 ± 6.73	2 (10.00%)	3 (15.00%)	15 (75.0%)
*t/χ* ^2^	0.740		0.314		1.112	
*P*	0.864		0.816		0.892	

**Table 2:** Univariate analysis of prognosis in patients with MM.

Factor	Survival (*n* = 61)	Death (*n* = 19)	*χ* ^2^	*P*
Gender			0.373	0.542
Male	37 (60.66%)	13 (68.42%)		
Female	24 (39.34%)	6 (31.58%)		

Age (years)			0.370	0.543
≥60	21 (34.43%)	8 (42.11%)		
<60	40 (65.57%)	11 (57.89%)		

DS staging			0.964	0.618
I	6 (9.84%)	3 (15.79%)		
II	11 (18.03%)	2 (10.53%)		
III	44 (2.13%)	14 (73.68%)		

PT (s)	12.25 ± 1.04	14.93 ± 0.75	10.401	<0.001
APTT (s)	33.18 ± 4.99	39.04 ± 3.57	4.745	<0.001
FIB (g/L)	2.83 ± 0.65	2.65 ± 0.50	1.108	0.272
TT (s)	14.35 ± 3.74	15.19 ± 3.87	0.848	0.399
D-D (*μ*g/ml)	2.07 ± 1.41	0.81 ± 0.17	3.870	<0.001
PLT (×10^9^/L)	165.07 ± 36.07	175.80 ± 35.10	1.139	0.258

**Table 3:** Assignment for multivariate logistic regression analysis.

Factors	Variables	Assignment
PT (s)	*X*1	Continuous variable
APTT (s)	*X*2	Continuous variable
D-D (*μ*g/ml)	*X*3	Continuous variable

**Table 4:** Multifactor analysis of prognosis of MM patients.

Variables	*B*	SE	Wals	*P*	OR	95% CI
PT (s)	1.283	0.341	14.156	0.012	3.607	1.849–7.038
APTT (s)	0.952	0.492	3.744	0.084	2.591	0.988–6.796
D-D (*μ*g/ml)	0.973	0.516	3.556	0.109	2.645	0.962–7.274

## Data Availability

The data can be obtained from the author upon reasonable request.
